This article has been retracted.

# SLCO4A1‐AS1 promotes cell growth and induces resistance in lung adenocarcinoma by modulating miR‐4701‐5p/NFE2L1 axis to activate WNT pathway

**DOI:** 10.1002/cam4.3270

**Published:** 2020-08-06

**Authors:** Yuxuan Wei, Li Wei, Jiwei Li, Zeheng Ma, Quan Zhang, Zhijun Han, Saisai Li

**Affiliations:** ^1^ Lanzhou University Second Hospital Lanzhou University Second Clinical Medical College Lanzhou China; ^2^ Department of Thoracic Surgery Henan Provincial People’s Hospital Zhengzhou University People’s Hospital Zhengzhou China

**Keywords:** chemosensitivity, lung adenocarcinoma, miR‐4701‐5p, NFE2L1, SLCO4A1‐AS1

## Abstract

Long noncoding RNAs (lncRNAs) possessed essential functions in the biological behaviors of various human cancers. SLCO4A1 antisense RNA 1 (SLCO4A1‐AS1) is a lncRNA that has been reported as a oncogenic regulator in colorectal cancer and bladder cancer. However, whether it exerted functions in the gene expression and cellular processes in lung adenocarcinoma (LUAD) remains still obscure. In the present research, we unveiled the high level of SLCO4A1‐AS1 in LUAD tissues and cells. Moreover, functional assays indicated that SLCO4A‐AS1 facilitated LUAD cell proliferation, motility, and cisplatin‐resistance. Besides, mechanism investigation revealed that miR‐4701‐5p could interact with SLCO4A1‐AS1 and directly target to NFE2L1. The expression correlation between miR‐4701‐5p and SLCO4A1‐AS1 or NFE2L1 was found to be negative. Moreover, NFE2L1 was expressed at a same tendency with SLCO4A1‐AS1 in LUAD tissues and cells. In addition, it was confirmed that NFE2L1 was involved in SLCO4A1‐AS1‐mediated activation of WNT pathway. According to rescue assays, NFE2L1 could involve in SLCO4A1‐AS1‐mediated LUAD cell growth. Conclusively, our study demonstrated that SLCO4A1‐AS1 facilitated cell growth and enhanced the resistance of LUAD cells to chemotherapy via activating WNT pathway through miR‐4701‐5p/NFE2L1 axis.

## Graphical abstract

Down‐regulation of SLCO4A1‐AS1 inhibits LUAD cell growth and promotes chemosensitivity. Up‐regulated SLCO4A1‐AS1 promotes LUAD cell growth and inhibits chemosensitivity. SLCO4A1‐AS1 acts as miR‐4701‐5p sponge in LUAD cells..

## 1 INTRODUCTION

Lung cancer is one of the leading causes of cancer‐associated deaths worldwide.^1^ Nonsmall cell lung cancer (NSCLC) is known as the main subtypes of lung cancer, among which, lung adenocarcinoma (LUAD) is a inducer of the high incidence rate and mortality. Great effort has been made in the therapeutic methods, such as chemotherapy, whereas late diagnosis and tumor metastasis lead to the low treatment efficiency.^2^ Cisplatin is a common chemotherapeutic agent using for solid tumors.^3^ Nevertheless, the efficiency of cisplatin to tumors is limit due to the chemoresistance in the late stage.^4^ Therefore, it is of great importance to decipher molecular mechanisms underneath the progression and chemoresistance of LUAD.

Long noncoding RNAs (LncRNAs), with length over 200 nucleotides, are considered as a cluster of transcripts without protein‐encoding ability, which are identified as the essential regulators in the initiation and progress of cancers.^5^ LncRNAs are involved in diverse cellular biological processes.^6^ Recently, studies have shown that LINC00673, HIT, HOTAIR, GAS5‐AS1, ANRIL, and PVT1, are crucial functional lncRNAs in the tumorigenesis of lung cancer.^7^ Moreover, the clinical relevance and underlying mechanisms of some lncRNAs have been elucidated in LUAD.^8^, ^9^ Although the functions of lncRNAs have been reported in LUAD, the specific mechanisms underlying their functions are largely marked. In consequence, it is in an urgent need to probe the underlying regulatory mechanisms of lncRNAs in LUAD. LncRNA SLCO4A1 antisense RNA 1 (SLCO4A1‐AS1) has been reported as an oncogene in colorectal cancer,^10^ whereas it has not been studied in LUAD.

Here, we aimed at deciphering the functional role and regulatory mechanism of SLCO4A1‐AS1 in LUAD cell growth and chemosensitivity.

## 2 MATERIALS AND METHODS

### 2.1 Tissue samples

A total of 40 pairs of LUAD tissues and normal tissues were obtained from patients from our hospital. All participants had not received any treatment before surgical resection. The written informed consent has been signed by all participants. Tissue samples used in this study were frozen in liquid nitrogen and then stored at −80°C as soon as surgical resection. Clinical study had been approved by the Ethics committee of our hospital.

### 2.2 Cell culture and treatment

LUAD cell lines (PC‐9, Calu3, A549, and HCC827) and human normal lung epithelial cell (BEAS‐2B) were available from ATCC (Manassas, VA), were preserved in a humidified incubator of 5% CO_2_ at 37. DMEM culture medium supplied with 1% antibiotics and 10% FBS (all, Gibco, Grand Island, NY) were used for cell culture. WNT pathway agonist LiCl (20 mM) was obtained from Sigma‐Aldrich (St. Louis, MI).

### 2.3 Total RNA extraction, cDNA synthesis, and qRT‐PCR

According to the standard methodology, TRIzol reagent (Thermo Fisher Scientific, Waltham, MA) was used for total RNA extraction. Reverse transcription was made using reverse Transcription Kit (Thermo Fisher Scientific) to synthesize cDNA. Afterward, PCR reaction system was prepared on Step‐One Plus Real‐Time PCR System (Applied Biosystems, Carlsbad, CA). GAPDH/U6 was regarded as the internal reference; the 2^−ΔΔCt^ method was applied for calculating relative gene expression. Primers used in this experiment were listed as follows: SLCO4A1‐AS1, Forward, 5′‐GGACATGCCGGTGATGAGAG‐3′; Reverse, 5′‐GACGCAGGGGTTCAAGTCAG‐3′; miR‐4701‐5p, Forward, 5′‐ATGAGTTGGCCACCACACCTA‐3′, Reverse, TTGGCCACCACACCTACCCCTT; NFE2L1, Forward, 5′‐GTGTGAACCTGGGAGTGCTT‐3′; Reverse, 5′‐ATTCAAAGTGGGGAAAAAGTGC‐3′; GAPDH, Forward, 5′‐CTCTGCTCCTCCTGTTCGAC‐3′; Reverse, 5′‐GCGCCCAATACGACCAAATC‐3′; U6, Forward, 5′‐CTCGCTTCGGCAGCACA‐3′; Reverse, 5′‐AACGCTTCACGAATTTGCGT‐3′. Each experimental procedure was repeated at least in triplicate.

### 2.4 Transfection

PC9 and A549 cells were seeded and incubated in 6‐well plates for 48 hours after transfected with indicated plasmids using Lipofectamine2000 (Invitrogen, Carlsbad, CA). The shRNAs and sh‐NC designed for SLCO4A1‐AS1, pcDNA3.1/NFE2L1, and pcDNA3.1 empty vector, miR‐4701‐5p mimics/inhibitor and corresponding controls NC mimics/inhibitor, were all procured from Genepharma (Shanghai, China) for gene silencing or overexpression. The target sequences of sh‐SLCO4A1‐AS1#1 or sh‐SLCO4A1‐AS1#2 were, respectively, as follow: 5′‐GTGCCTTGCAGAGCTGATGTT‐3′ and 5′‐GACCTCAGCAGCCATGAACAT‐3′. Each experimental procedure was repeated at least in triplicate.

### 2.5 Colony formation

PC9 and A549 cells were transplanted into 6‐well plates at 37°C with 5% CO_2_ for 14 days. After washing in PBS, 1 mL of 0.1% crystal violet was added for staining, and then colonies with over 50 cells were counted. Each experimental procedure was repeated at least in triplicate.

### 2.6 EdU assay

To assess cell proliferation ability, transfected LUAD cells cultured in 96‐well plates were treated with EdU assay kit (Ribobio, Guangzhou, China). Following staining of cell nuclei with Hoechst 33342 solution, EdU‐stained cells were monitored by fluorescent microscope. Each experimental procedure was repeated at least in triplicate.

### 2.7 Caspase‐3 activity test

Caspase‐3 Activity Kit was available from Solarbio (Beijing, China). Protein extracts obtained from transfected cells were planted in 96‐well plates adding caspase‐3 substrate and reaction buffer at 37°C. Four hours later, caspase‐3 activity was determined at 405 nm through microplate reader. Each experimental procedure was repeated at least in triplicate.

### 2.8 TUNEL assay

Cell apoptosis was also detected with the application of TUNEL assay kit (Beyotime, Shanghai, China) as per specific direction. After dying cell nucleus with DAPI, TUNEL‐stained cell samples were determined under fluorescent microscope. Each experimental procedure was repeated at least in triplicate.

### 2.9 Wound‐healing assay

Transfected LUAD cells were cultured in 6‐well plates were until the confluence reached to 90%. Following replacing culture medium with serum‐free medium, the single cell layer was scratched with 10 μL pipette tip. Images of migrated cells were observed at 0 and 24 hours under a microscope. Each experimental procedure was repeated at least in triplicate.

### 2.10 Transwell invasion assay

LUAD cells (2 × 10^3^) cultured in serum‐free medium were seeded in upper transwell chambers with Matrigel‐coated (BD Biosciences, Franklin Lakes, NJ). Complete culture medium was added to lower chamber. Invasive cells were processed with 0.1% crystal violet staining solution for 15 minutes, and then counted under microscope. Each experimental procedure was repeated at least in triplicate.

### 2.11 MTT assay

PC9 and A549 cells were transfected for 48 hours, then collected to treat in 96‐well plates with cisplatin (Sigma‐Aldrich) at various concentrations. To assess the IC_50_ concentration of cisplatin, 20 μL of MTT (0.5 mg/mL; Sigma‐Aldrich) was added for 4 hours. After adding 200 μL of DMSO (Sigma‐Aldrich), the absorbance at 490 nm was examined by microplate reader. Each experimental procedure was repeated at least in triplicate.

### 2.12 Subcellular fractionation

Using PARIS™ Kit (Ambion, Austin, TX), nucleus or cytoplasm of PC9 and A549 cells were acquired in accordance with the manual. Isolated RNAs were detected by qRT‐PCR, using GAPDH and U6 as the cytoplasmic or nuclear control. Each experimental procedure was repeated at least in triplicate.

### 2.13 FISH

For FISH assay, 6 × 10^4^ cells were planted into each well of 24‐well plates. According to the protocol of FISH kit (C10910, Ribobio, Guangzhou, Guangdong, China), FISH assay was conducted when the confluence reached to 60%‐70%. LUAD cells were then fixed with 4% paraformaldehyde and permeated with 0.5% Triton X‐100 solution at 4°C SLCO4A1‐AS1‐FISH probe was designed and produced by Ribobio in line with the manual. Fixed cells in 4% formaldehyde were air‐dried and hybridized with RNA FISH probe, followed by Hoechst staining for nuclear detection. Stained cells were finally observed by a fluorescent microscope (DMI8, Leica, Mannheim, Germany). Each experimental procedure was repeated at least in triplicate.

### 2.14 RNA immunoprecipitation (RIP)

RIP experiments were performed via utilizing EZ‐Magna RIP™ RNA Binding Protein Immunoprecipitation Kit (17‐701, Millipore). In brief, the isolated LUAD cells were rinsed in PBS, trypsinized, and centrifuged for RIP assay. Afterward, cells were lysed with RIP buffer supplemented with RNase inhibitor. RIP buffer containing magnetic beads conjugated with Ago2 antibody was used to incubate 100 μL of whole cell extract. Input containing 10% cell lysates acted as the positive control and antibodies targeting IgG were the negative control. Besides, RNAs precipitated in these three groups were also subjected to qRT‐PCR. Each experimental procedure was repeated at least in triplicate.

### 2.15 RNA pull down

The Pierce Magnetic RNA‐Protein Pull‐Down Kit (Thermo Fisher Scientific, Waltham, MA, USA) was utilized for RNA pull‐down assay. SLCO4A1‐AS1 sequence was labeled with biotin probe. SLCO4A1‐AS1 sequence without biotin label was used as the negative control. Subsequently, cell lysates were incubated with biotin‐SLCO4A1‐AS1 probe or nonbiotin probe following with the incubation of the magnetic beads for 30 minutes. Finally, the complex was washed and RNAs were purified with TRIzol reagent (Thermo Fisher Scientific). qRT‐PCR analysis was used to detect RNA enrichment in two groups. Each experimental procedure was repeated at least in triplicate.

### 2.16 Luciferase reporter assay

The SLCO4A1‐AS1 or NFE2L1 fragments, covered wild‐type and mutated‐binding sites of miR‐4701‐5p, were inserted into pmirGLO vector (Promega, Madison, WI), termed SLCO4A1‐AS1‐WT/Mut and NFE2L1‐WT/Mut. After co‐transfection with miR‐4701‐5p mimics or NC mimics, Luciferase Reporter Assay System (Promega) was applied to assess luciferase activity. Besides, the TOP‐flash and FOP‐flash vectors were available from Addgene (Cambridge, MA) to measure Wnt/β‐catenin signaling using luciferase assay. Each experimental procedure was repeated at least in triplicate.

### 2.17 Western blot

The total proteins from LUAD cells were electrophoresed by 10% SDS‐PAGE, then loaded to the PVDF membranes and blocked with 5% nonfat milk powder. The primary antibodies against NFE2L1, β‐catenin, CDK1, MYC, AXIN2, SOX4, MMP2, and GAPDH were obtained from Abcam (Cambridge, MA, USA), along with the corresponding secondary antibody. After washing, enhanced chemiluminescence reagent (Santa Cruz Biotechnology, Santa Cruz, CA, USA) was used to detect band density. Each experimental procedure was repeated at least in triplicate.

### 2.18 Tumor growth in nude mice

Nude mice were purchased from National Laboratory Animal Center (Beijing, China). Transfected PC9 cells were subcutaneously injected into the axilla of nude mice. Four weeks later, the mice were sacrificed. Then, tumors were excised and weighed. Volume was measured as length × width^2^ × 0.5. The experiment was approved by the Ethics Committee for Animal Research of hospital.

### 2.19 Statistical analyses

Each experiment included more than three various bio‐replications. Results were all displayed with standard deviation. Pearson correlation analysis was applied to evaluate the correlation between NFE2L1 expression and SLCO4A1‐AS1 expression. Graphpad Prism 6 software was applied for data analysis with Student's *t* test and one‐way or two‐way ANOVA, with *P*‐values below .05 indicated statistical significance.

## 3 RESULTS

### 3.1 Downregulation of SLCO4A1‐AS1 inhibits LUAD cell growth and promotes chemosensitivity

First, we detected SLCO4A1‐AS1 expression in LUAD tissues and adjacent normal tissues. SLCO4A1‐AS1 was significantly upregulated in LUAD tissues than that in adjacent normal tissues (Figure 1A). Then, SLCO4A1‐AS1 expression in LUAD cell lines (PC‐9, Calu3, A549, and HCC827) and human normal lung epithelial cell (BEAS‐2B) was assessed via qRT‐PCR. As a result, SLCO4A1‐AS1 was notably overexpressed in LUAD cells, especially in PC‐9 and A549 cells (Figure 1B). To decipher the function of SLCO4A1‐AS1 in LUAD cells, SLCO4A1‐AS1 expression was stably silenced in PC‐9 and A549 cells (Figure S1A). Through colony formation and EdU assays, we observed that the proliferative ability of PC‐9 and A549 cells was considerably impaired upon SLCO4A1‐AS1 depletion (Figure 1C and D). In addition, the apoptosis in sh‐SLCO4A1‐AS1 transfected PC‐9 and A549 cells was significantly increased in comparison of sh‐NC group (Figure 1E and F). Wound healing assay manifested that SLCO4A1‐AS1 knockdown in PC‐9 and A549 cells led to an evident suppression in the migration (Figure 1G). Based on transwell assay, the invasive capacity of PC‐9 and A549 cells was alleviated by the silencing of SLCO4A1‐AS1 (Figure 1H). MTT assay implied that the decreased viability in cisplatin‐treated cells was more evident after silencing of SLCO4A1‐AS1 than sh‐NC group, and IC_50_ concentration of cisplatin was decreased by SLCO4A1‐AS1 deficiency (Figure 1I).

**FIGURE 1:** Downregulation of SLCO4A1‐AS1 inhibits LUAD cell growth and promotes chemosensitivity. (A and B) qRT‐PCR assessed SLCO4A1‐AS1 expression in LUAD tissues and control normal tissues, as well as in LUAD cells (PC‐9, Calu3, A549, and HCC827) and human normal lung epithelial cell (BEAS‐2B). (C and D) The proliferation in sh‐SLCO4A1‐AS1 transfected cells was determined by colony formation and EdU assay (scale bar = 100 μm). (E and F) Caspase‐3 activity assay and TUNEL assay (scale bar = 100 μm) were conducted for detecting cell apoptosis upon SLCO4A1‐AS1 knockdown. (G) The migratory ability of PC‐9 and A549 cells transfected with sh‐SLCO4A1‐AS1 was validated by wound healing assay (scale bar = 100 μm). (H) Transwell assay (scale bar = 100 μm) was carried out to confirm the invasion of SLCO4A1‐AS1 silenced PC‐9 and A549 cells. (I) Effect of silenced SLCO4A1‐AS1 on cell chemosensitivity to cisplatin was confirmed via MTT assay. ^*^ *P* < .05, ^**^ *P* < .01

Meanwhile, the function of SLCO4A1‐AS1 overexpression in LUAD cell proliferation, migration, invasion, and cisplatin sensitivity was examined. The overexpression of SLCO4A1‐AS1 induced by pcDNA3.1‐SLCO4A1‐AS1 was verified by qRT‐PCR assay (Figure 2A). Then, colony formation and EdU assay revealed that overexpression of SLCO4A1‐AS1 enhanced cell proliferation (Figure 2B and C). Wound healing and transwell invasion assay disclosed that cell migration and invasion ability were elevated by SLCO4A1‐AS1 overexpression (Figure 2D and E). Besides, upregulated SLCO4A1‐AS1 decreased the sensitivity to cisplatin (Figure 2F). Taken all together, SLCO4A1‐AS1 promotes LUAD cell growth, motility, and chemoresistance.

**FIGURE 2:** Upregulated SLCO4A1‐AS1 promotes LUAD cell growth and inhibits chemosensitivity. (A) qRT‐PCR revealed SLCO4A1‐AS1 expression in cells transfected with pcDNA3.1‐SLCO4A1‐AS1. (B and C) Cell proliferation in pcDNA3.1‐SLCO4A1‐AS1 transfected cells was determined by colony formation and EdU assay (scale bar = 100 μm). (D) The migratory ability of PC‐9 and A549 cells transfected with pcDNA3.1‐SLCO4A1‐AS1 was validated by wound healing assay (scale bar = 100 μm). (E) Transwell assay (scale bar = 100 μm) was carried out to confirm the invasion of PC‐9 and A549 cells by upregulation of SLCO4A1‐AS1. (F) The IC_50_ values of cisplatin in cisplatin‐resistant PC9 and A549 cells were determined by MTT assay. ^**^ *P* < .01

### 3.2 SLCO4A1‐AS1 acts as miR‐4701‐5p sponge in LUAD cells

Results of subcellular fractionation and FISH assays showed the abundant expression of SLCO4A1‐AS1 in the cytoplasm (Figure 3A and B), suggesting that SLCO4A1‐AS1 might modulate the expressions of downstream genes at the post‐transcriptional level. RIP assay showed that SLCO4A1‐AS1 could bind to RNA‐induced silencing complexes (RISCs), which indicated that SLCO4A1‐AS1 might function as a ceRNA (Figure 3C). Using DIANA database (http://diana.imis.athena‐innovation.gr/DianaTools/index.php?r=tarbase/index), 14 miRNAs (score >0.8) were predicted to be the potential downstream RNAs of SLCO4A1‐AS1 (Figure 3D). Then, the expressions of predicted miRNAs were detected in LUAD cells and BEAS‐2B cell. The results indicated that six miRNAs were differentially expressed in LUAD cells, among which, four miRNAs (miR‐149‐5p, miR‐4304, miR‐4283, and miR‐876‐3p) were upregulated and two miRNAs (miR‐4701‐5p and miR‐5001‐3p) were downregulated (Figure 3E). Therefore, miR‐4701‐5p and miR‐5001‐3p were selected for further analysis. RNA pull‐down assay displayed that miR‐4701‐5p was obviously enriched in the SLCO4A1‐AS1 biotin probe (Figure 3F). In addition, miR‐4701‐5p showed a low level in LUAD tissues and cells compared with normal control tissues and cells (Figure 3G). RIP assay delineated that both SLCO4A1‐AS1 and miR‐4701‐5p were remarkably enriched in Ago2 immunoprecipitation (Figure 3H). Then, miR‐4701‐5p was overexpressed in PC‐9 and A549 cells (Figure S1B), and the putative binding site of miR‐4701‐5p on SLCO4A1‐AS1 sequence was illustrated and a mutation was produced (Figure 3I). As expected, miR‐4701‐5p overexpression suppressed the luciferase activity of wild‐type SLCO4A1‐AS1 (Figure 3J). Collectively, SLCO4A1‐AS1 acts as miR‐4701‐5p sponge in LUAD cells.

**FIGURE 3:** SLCO4A1‐AS1 acts as miR‐4701‐5p sponge in LUAD cells. (A and B) The distribution of SLCO4A1‐AS1 was certificated through subcellular fractionation assay and FISH assay (scale bar = 100 μm). (C) RIP assay confirmed the interaction of SLCO4A1‐AS1 with RISCs. (D) The potential miRNAs that could bind to SLCO4A1‐AS1 were obtained from DIANA. (E) Expression differences of predicted miRNAs in LUAD cells. (F) RNA pull‐down assay was performed for screening the potential miRNAs for SLCO4A1‐AS1. (G) MiR‐4701‐5p expression level in LUAD tissues and cells compared to normal tissues and cells was evaluated by qRT‐PCR. (H) The enrichments of SLCO4A1‐AS1 and miR‐4701‐5p in the beads conjugated with Ago2 antibody were determined by RIP assay. (I) Putative miR‐4701‐5p binding site to SLCO4A1‐AS1. (J) The binding between SLCO4A1‐AS1 and miR‐4701‐5p was assessed via performing luciferase reporter assay. ^*^ *P* < .05, ^**^ *P* < .01

### 3.3 NFE2L1 is a target gene of miR‐4701‐5p

Subsequently, we applied three databases (RNA22, miRmap, and microT) to screen out target genes for miR‐4701‐5p, and 5 mRNAs (DDI2, NT5DC3, NFE2L1, ZFHX3, and RANBP10) were predicted (Figure 4A). Through the results of qRT‐PCR, NFE2L1 was found to be upregulated in LUAD cells, whereas other mRNAs showed no significant differences (Figure 4B). Therefore, NFE2L1 was selected for further study. Then, we fund that NFE2L1 was significantly overexpressed in LUAD tissues and had a positive correlation with SLCO4A1‐AS1 in 40 LUAD tissues (Figure 4C). Furthermore, the mRNA and protein levels of NFE2L1 were significantly decreased in PC‐9 and A549 cells transfected with miR‐4701‐5p mimics or sh‐SLCO4A1‐AS1 (Figure 4D and E). Besides, RIP assay depicted the observable enrichment of SLCO4A1‐AS1, miR‐4701‐5p, and NFE2L1 in the beads conjugated with Ago2 antibody (Figure 4F). It was displayed that NFE2L1 3'UTR contains a potential miR‐4701‐5p‐binding site (Figure 4G). Luciferase reporter assay indicated that luciferase activity in NFE2L1‐WT group was notably lessened by the overexpression of miR‐4701‐5p (Figure 4H). Then, the transfection efficiency of miR‐4701‐5p inhibitor was detected, and results demonstrated the decreased miR‐4701‐5p expression in cells transfected with miR‐4701‐5p inhibitor (Figure S1C). In addition, inhibited NFE2L1 expression in PC‐9 and A549 cells caused by SLCO4A1‐AS1 knockdown was restored by the inhibition of miR‐4701‐5p (Figure 4I). All the data suggested that NFE2L1 is a target gene of miR‐4701‐5p.

**FIGURE 4:** NFE2L1 is a target gene of miR‐4701‐5p. (A) Predicted target genes of miR‐4701‐5p. (B) Expressions of predicted mRNAs in LUAD cells (PC‐9, Calu3, A549, and HCC827) and human normal lung epithelial cell (BEAS‐2B). (C) NFE2L1 expression in clinical tissue was assessed by qRT‐PCR; the correlation between NFE2L1 expression and SLCO4A1‐AS1 expression in 40 LUAD tissues was evaluated by Pearson's correlation analysis. (D) NFE2L1 expression in PC‐9 and A549 cells transfected with miR‐4701‐5p mimics was evaluated by qRT‐PCR and western blot assay. (E) Effect of silenced SLCO4A1‐AS1 on NFE2L1 expression was evaluated by qRT‐PCR and western blot assay. (F) RIP assay was carried out for testing the enrichment of SLCO4A1‐AS1, miR‐4701‐5p, and NFE2L1. (G) Predicted miR‐4701‐5p binding site on SLCO4A1‐AS1. (H) Luciferase reporter assay was employed for evaluating the combination between miR‐4701‐5p and NFE2L1. (I) sh‐NC, sh‐SLCO4A1‐AS1, sh‐SLCO4A1‐AS1 + miR‐4701‐5p inhibitor were transfected into PC‐9 and A549 cells, and then NFE2L1 expression was detected by qRT‐PCR and western blot assay. ^**^ *P* < .01

### 3.4 NFE2L1 restores the suppressive effects of SLCO4A1‐AS1 on WNT pathway in LUAD cells

SLCO4A1‐AS1 has been reported to activate WNT pathway in colorectal cancer.^10^ Here, we wondered whether NFE2L1 was involved in SLCO4A1‐AS1‐activated WNT pathway in LUAD. At first, NFE2L1 expression was elevated by transfection of pcDNA3.1/NFE2L1 (Figure S1D). Then, we classified the experiments into three groups: sh‐NC, sh‐SLCO4A1‐AS1#1, sh‐SLCO4A1‐AS1#1 + pcDNA3.1/NFE2L1. Next, TOP/FOP assay was performed to determine the activity of WNT pathway. The results expound that overexpressed NFE2L1 counteracted the inhibitory influence of SLCO4A1‐AS1 on WNT pathway activity (Figure 5A). Through subcellular fractionation assay, we observed that nuclear translocation of β‐catenin (CTNNB1) was repressed by silenced SLCO4A1‐AS1, but was further promoted via co‐transfection of pcDNA3.1‐NFE2L1 (Figure 5B). Furthermore, the mRNA and protein levels of NFE2L1 and WNT pathway‐related genes (CDK1, AXIN2, SOX4, MYC, and MMP2) were all reduced in sh‐SLCO4A1‐AS1 transfected cells, but were further elevated by co‐transfection of pcDNA3.1‐NFE2L1 (Figure 5C and D). WNT pathway activator (LiCl) was further used to perform rescue assays. Through EdU assay, the treatment of LiCl reserved the suppressed proliferation in cells transfected with sh‐SLCO4A1‐AS1 (Figure 5E). In addition, the enhanced apoptosis caused by SLCO4A1‐AS1 depletion was offset by treating with LiCl (Figure 5F). All results elucidated that SLCO4A1‐AS1 activates WNT pathway via upregulation of NFE2L1 in LUAD cells.

**FIGURE 5:** SLCO4A1‐AS1‐activated WNT pathway in LUAD via NFE2L1. (A) The activity of WNT pathway was determined by TOP/FOP assay. (B) The nuclear translocation of β‐catenin (protein form of CTNNB1) was analyzed via subcellular fractionation assay. (C) Expression of NFE2L1 and WNT pathway‐related genes was analyzed by qRT‐PCR in indicated PC‐9 and A549 cells. (D) NFE2L1 protein and WNT pathway‐related proteins were examined by western blot assay. (E and F) The proliferation and apoptosis were tested in the cells transfected with sh‐NC, sh‐SLCO4A1‐AS1, and sh‐SLCO4A1‐AS1 + LiCl by EdU and TUNEL assays. ^**^ *P* < .01

### 3.5 SLCO4A1‐AS1 enhances LUAD progression by upregulating NFE2L1

Finally, we explored whether SLCO4A1‐AS1 enhanced LUAD cell growth by regulating NFE2L1 by conducting some rescue assays. Results from colony formation and EdU assays disclosed that depleted SLCO4A1‐AS1 markedly restrained the proliferation in LUAD cells but the transfection of pcDNA3.1/NFE2L1 recovered this effect (Figure 6A and B). In addition, cell apoptosis increased by SLCO4A1‐AS1 deficiency was restored by NFE2L1 overexpression (Figure 6C and D). Besides, overexpressed NFE2L1 countervailed the sh‐SLCO4A1‐AS1‐mediated alleviation on migration and invasion (Figure 6E and F). Overexpressed NFE2L1 counteracted the repressive influence of silenced SLCO4A1‐AS1 on cell resistance to cisplatin (Figure 6G). Moreover, the mice model was established to evaluate the functional role of SLCO4A1‐AS1/NFE2L1 axis in‐vivo. The tumor photos were shown in Figure 6H. Tumor volume and weight were reduced by silenced SLCO4A1‐AS1, whereas upregulated NFE2L1 neutralized the suppressive effects of inhibited SLCO4A1‐AS1 on tumor volume and weight (Figure 6I). In brief, SLCO4A1‐AS1 enhances LUAD progression by upregulating NFE2L1.

**FIGURE 6:** slco4a1‐as1 enhances luad progression by upregulating nfe2l1. (A and B) The proliferation of sh‐NC, sh‐SLCO4A1‐AS1, and sh‐SLCO4A1‐AS1 + pcDNA3.1/NFE2L1 transfected cells was evaluated by colony formation and EdU assay (scale bar = 100 μm). (C and D) The apoptosis of PC‐9 and A549 cells transfected with sh‐NC, sh‐SLCO4A1‐AS1, and sh‐SLCO4A1‐AS1 + pcDNA3.1/NFE2L1 was tested via caspase‐3 activity assay and TUNEL assay (scale bar = 100 μm). (E and F) Role of sh‐NC, sh‐SLCO4A1‐AS1, and sh‐SLCO4A1‐AS1 + pcDNA3.1/NFE2L1 plasmids in cell migration and invasion was measured through wound healing (scale bar = 100 μm) and transwell assays (scale bar = 100 μm). (G) The IC_50_ value of cisplatin in PC9 cells by indicated transfections was determined by MTT assay. (H) Photos of tumor obtained from nude mice after injection of different transfected cells. (I) Tumor volume and weight in different groups. ^**^ *P* < .01

## 4 DISCUSSION

LUAD is a malignant cancer with unfavorable outcome. The unsatisfied prognosis of LUAD is closely associated with the activation of metastasis and invasion.^11^ Abnormal expressions of cancer‐related gene exhibit the pivotal functional roles in LUAD progression. It has been confirmed that a large number of genomes are transcribed as noncoding RNAs, mainly as lncRNAs and microRNAs (miRNAs).^12^ A variety of lncRNAs were validated to modulate target genes expressions via diverse mechanisms.^13^ In recent years, increasing studies have elucidated that the dysregulation of lncRNAs participated in multiple biological behaviors and played crucial roles in LUAD tumor initiation and development.^14^ LncRNA SLCO4A1‐AS1 has been reported to drive colorectal cancer cell growth by activating Wnt pathway.^10^ Furthermore, SLCO4A1‐AS1 was reported to promote cell invasion and upregulate OCT4 expression through sponging miR‐335‐5p in bladder cancer.^15^ However, the role of SLCO4A1‐AS1 has not been revealed in LUAD. In this study, it was discovered that SLCO4A1‐AS1 was highly expressed in LUAD cells, and the silencing of SLCO4A1‐AS1 hampered cell proliferation, migration and invasion, induced cell apoptosis, and promoted chemosensitivity. These results presented the oncogenic property of SLCO4A1‐AS1 in LUAD cell growth.

MiRNAs are about 21‐24 nucleotides in length, which can lead to the degradation or translation inhibition of target mRNAs via targeting its 3′‐UTRs.^16^ One of the common mechanisms of lncRNAs is that lncRNAs combine with miRNAs to modulate its target genes by acting as competing endogenous RNA (ceRNA).^17^ For example, SNHG6 upregulates E2F7 and promotes epithelial mesenchymal transition (EMT) and proliferation via sponging miR‐26‐5p in LUAD.^18^ LncRNA MIAT promotes metastasis and cell growth in gastric cancer growth via regulating miR‐141/DDX5 axis.^19^ The interaction of lncRNAs with miRNAs exhibited important roles in the regulation of biological behaviors of malignant tumors. Hence, it is beneficial to further explore this interaction for improving the treatment efficacy of LUAD.

MiR‐4701‐5p has been studied in chronic myeloid leukemia, but its functions and mechanism in LUAD, is rarely elucidated. Here, we found that miR‐4701‐5p was downregulated in LUAD cells and sponged by SLCO4A1‐AS1. Furthermore, NFE2L1 was identified as the target gene of miR‐4701‐5p and was upregulated in LUAD cells. WNT pathway is a classical pathway which has been widely reported in cancers, and its dysregulation is strongly associated with tumor progression.^20^ Our study manifested that SLCO4A1‐AS1 knockdown effectively decreased the activity of WNT pathway, inhibited nuclear translocation of β‐catenin, and suppressed the expression of WNT pathway‐relevant genes. Previously, studies have unveiled that the motif of NFE2L1 (also referred to as NRF1) was enriched in several genes involved in WNT signaling pathway in breast cancer.^21^ However, it seemed that NFE2L1 was targeted by β‐catenin during endodermal differentiation based on the findings of a recent report.^22^ Presently, we discovered that NFE2L1 was implicated in the regulation of SLCO4A1‐AS1 on WNT pathway. Moreover, activation of WNT pathway via LiCl treatment recovered the inhibitory effect of SLCO4A1‐AS1 depletion on LUAD cell growth. Rescue assays suggested that the suppressive effect of SLCO4A1‐AS1 deficiency in LUAD cell functions was abolished by NFE2L1 overexpression.

In conclusion, this study revealed a novel highly expressed lncRNA SLCO4A1‐AS1 in LUAD. SLCO4A1‐AS1 promoted cell growth and inhibited chemosensitivity in LUAD via miR‐4701‐5p/NFE2L1 axis to stimulate WNT pathway, which might be helpful for deciphering novel therapeutic methods for LUAD patients.

## 5 ETHICS STATEMENT

The written informed consent has been signed by all participants. A total of 40 pairs of LUAD tissues and normal tissues were obtained from patients from the Lanzhou University Second Hospital. The experiment was approved by the Ethics Committee for Animal Research of the Lanzhou University Second Hospital.

## CONFLICTS OF INTERESTS

Authors state no conflicts of interest in this study.

## Supporting information


**Figure S1**

## Data Availability

Not applicable.
